The article "Clinical evaluation of new automatic coronary-specific best cardiac phase selection algorithm for single-beat coronary CT angiography" was published in 2017. Journal: PLoS One.

# Clinical evaluation of new automatic coronary-specific best cardiac phase selection algorithm for single-beat coronary CT angiography

**DOI:** 10.1371/journal.pone.0172686

**Published:** 2017-02-23

**Authors:** Hui Wang, Lei Xu, Zhanming Fan, Junfu Liang, Zixu Yan, Zhonghua Sun

**Affiliations:** 1 Department of Radiology, Beijing Anzhen Hospital, Capital Medical University, Beijing, China; 2 Department of Radiology, Beijing Huairou Hospital, Beijing, China; 3 Department of medical radiation Sciences, Curtin University, Perth, Western Australia, Australia; Universita degli Studi Magna Graecia di Catanzaro, ITALY

## Abstract

The aim of this study was to evaluate the workflow efficiency of a new automatic coronary-specific reconstruction technique (Smart Phase, GE Healthcare—SP) for selection of the best cardiac phase with least coronary motion when compared with expert manual selection (MS) of best phase in patients with high heart rate. A total of 46 patients with heart rates above 75 bpm who underwent single beat coronary computed tomography angiography (CCTA) were enrolled in this study. CCTA of all subjects were performed on a 256-detector row CT scanner (Revolution CT, GE Healthcare, Waukesha, Wisconsin, US). With the SP technique, the acquired phase range was automatically searched in 2% phase intervals during the reconstruction process to determine the optimal phase for coronary assessment, while for routine expert MS, reconstructions were performed at 5% intervals and a best phase was manually determined. The reconstruction and review times were recorded to measure the workflow efficiency for each method. Two reviewers subjectively assessed image quality for each coronary artery in the MS and SP reconstruction volumes using a 4-point grading scale. The average HR of the enrolled patients was 91.1±19.0bpm. A total of 204 vessels were assessed. The subjective image quality using SP was comparable to that of the MS, 1.45±0.85 vs 1.43±0.81 respectively (p = 0.88). The average time was 246 seconds for the manual best phase selection, and 98 seconds for the SP selection, resulting in average time saving of 148 seconds (60%) with use of the SP algorithm. The coronary specific automatic cardiac best phase selection technique (Smart Phase) improves clinical workflow in high heart rate patients and provides image quality comparable with manual cardiac best phase selection. Reconstruction of single-beat CCTA exams with SP can benefit the users with less experienced in CCTA image interpretation.

## Introduction

Coronary computed tomography angiography (CCTA) plays an important role in coronary artery disease management, especially for exclusion of significant coronary artery stenosis because of the test’s high negative predictive value [1–3]. It often serves as the gatekeeper to invasive diagnostic and surgical procedures [4]. The accuracy of diagnostic interpretation by CCTA highly depends on good reconstruction image quality, since the cardiac motion artifacts may compromise the diagnostic image quality. Often times, multiple segments of the cardiac cycle are acquired based on the heart rate due to the fact that the quiescent cardiac phase with the least coronary motion within this cycle is dependent, in part, on this heart rate. Recent developments of multi-slice CT scanner make it possible to acquire abundant data with excellent temporal and spatial resolution with a short scan time [5–7]. However, it is a time-consuming process for radiologists or medical imaging technologists to pick up the best phase with the least motion from the phase of the cardiac cycle for reconstruction, in particular this presents a challenge for newer users of the technology in clinical centers with large patient volumes, and in clinical settings where CT imaging is done even in the presence of higher heart rates. Thus, it would be useful to find an automatic way to determine the best phase of the cardiac cycle for CCTA reconstruction.

The article "Clinical evaluation of new automatic coronary-specific best cardiac phase selection algorithm for single-beat coronary CT angiography" was published in 2017. Journal: PLoS One.

Recently, a brand new automated algorithm for selecting the optimal cardiac phase for CCTA reconstructions had been developed [8]. However, its clinical efficiency has not been evaluated. The objective of this study was to evaluate, in high heart rate patients, the performance and workflow efficiency of this new automatic coronary-specific cardiac phase selection reconstruction technique (Smart Phase, GE Healthcare) for selecting the best phase with least coronary motion compared with manual selection of the best phase by an expert.

## Materials and methods

### Patient selection

The Institutional Review Board of Beijing Anzhen Hospital approved this study. From April 2016 to May 2016, a total of 48 consecutive patients with heart rates above 75 bpm, who were referred to undergo CCTA were prospectively enrolled. Written informed consent was obtained from all patients. The exclusion criteria for CCTA were as follows: allergic to iodine-containing contrast medium, renal insufficiency (creatinine clearance of <60 mL/min per 1.73 m^2^), inability to follow breath-hold instructions. The patient who had undergone coronary revascularization, including percutaneous coronary interventions and coronary artery bypass graft were also excluded. Two patients were excluded because of prior coronary revascularizations. Thus, 46 patients (22 men, 24 women; mean age, 58.4±11.3 years; age range, 31–78 years) were enrolled in the study.

The article "Clinical evaluation of new automatic coronary-specific best cardiac phase selection algorithm for single-beat coronary CT angiography" was published in 2017. Journal: PLoS One.

### CCTA data acquisition

All CT examinations were performed on a 256 detector row CT scanner (Revolution CT, GE Healthcare, Waukesha, Wisconsin, US). The patients were instructed to practice breath holding before scanning. The contrast media were preheated in a heating box to 37°C before injection, and were applied using a dual-head power injector (Stellant; Medrad, Indianola, United States). The contrast medium was injected at an injection rate of 5 mL/s in all patients. The total contrast volume for each patient was 75 ml. All injections were followed by 30 ml of saline flush. The image acquisition was triggered after a threshold of 60 HU was reached in a region of interest placed in the ascending aorta (bolus-tracking technique). None of the patients received sublingual nitroglycerine. Data were acquired in craniocaudal direction. The scanning range was from the tracheal bifurcation to cardiac apex within single beat. All data were acquired with the following parameters: The slice thickness and interval for reconstruction were both 0.625 mm. 50% adaptive statistical iterative reconstruction (ASiR-V) was adopted. The reconstruction matrix was 512×512. The tube voltage was set using kV-assist, and the tube current was determined by using smart-mA, and the optional range was 200–650 mA. The preset noise index (NI) was 25 HU. The gantry rotation time was 0.28 s/rot. For the patients with a heart rate of 75–85 bpm, exposure windows was set at the 30%–80% RR intervals, while for those with a heart rate faster than 86 bpm, the exposure window was set at the 40–60% RR interval.

### Coronary CT angiography image reconstruction

Coronary CT angiography images were reconstructed with a slice thickness of 0.625 mm and the same increment, using standard kernel. After anonymization, reconstructions were performed at 5% phase intervals. An expert with more than 5 years’ experience in interpreting CCTA manually selected from these phases the “best” phase, with minimized coronary motion (MS). The time for reconstruction of each phase as well as the time to select the best phase were recorded. Separately, the phase selection (Smart Phase, GE Healthcare) algorithm was used to identify and reconstruct the algorithmically determined best phase (SP). And the reconstruction phase intervals of the SP were 2%. This algorithm works by applying coronary specific quantitative image quality (IQ) metrics during the reconstruction process to search and identify the phase of least coronary motion. Similar to MS, the reconstruction time (including processing by the phase selection algorithm) was recorded. If absolute phase were picked out as the best phase by either MS or SP, it would be changed into relative phase for statistical analysis.

The article "Clinical evaluation of new automatic coronary-specific best cardiac phase selection algorithm for single-beat coronary CT angiography" was published in 2017. Journal: PLoS One.

### Image analysis

The MS and SP images were transferred to a workstation (GE Advantage Workstation 4.6) for post-processing. Curved planar reformation (CPR) was generated for further analysis. Original two-dimensional transverse and curved planer reformation (CPR) images were used for assessment of image quality. Two radiologists, each with more than 5 years of experience in cardiovascular imaging, were blinded to the best phase selection methods and independently assessed the coronary arteries. Any discrepancy between the 2 reviewers was resolved during a third session, through which the reviewers read images together to reach a consensus. Image quality for each coronary artery was evaluated with a 4-point grading scale [9]. Segments that could not be evaluated (non-diagnostic) were given a score of 4, corresponding to poor vessel opacification, lack of vessel wall definition due to marked motion artifacts, severe image noise-related blurring. Segments that could be evaluated (being diagnostic) were scored as follows: A score of 3 corresponded to fair vessel opacification, some motion artifacts or noise-related blurring, or moderate structural discontinuity but sufficient delineation of the individual segments; a score of 2, good vessel opacification, minor motion artifacts or noise-related blurring, and minimal vessel discontinuity; and a score of 1, excellent vessel opacification, absence of motion artifacts or noise-related blurring, and no structural discontinuity. As each vessel has several segments, the segment with lowest score would be defined as a score of the corresponding vessel.

### Statistical analysis

Quantitative variables were expressed as mean ± SD, and categorical variables were expressed as frequencies or percentages. The reconstruction time was compared between the 2 groups by using the Student t test. The Wilcoxon signed rank test was used to evaluate the difference in the subjective image quality between best phase selection techniques. The total vessels as well as the individual coronary arteries, including right coronary artery (RCA) and its branches posterior decending artery (PDA), left anterior decending artery (LAD) and its branches diagonal branch (D), left circumflex artery (LCX) and its branches obtuse marginal branch (OM), were evaluated sepreately. We assessed the difference in phases between the two techniques using chi-square test and Bland-Altman analysis. Box-plot analysis was used to assess rater distributional differences. Inter-observer agreement in subjective image quality assessment was evaluated by κappa statistics. A κ value of 0 indicates poor agreement; 0.01 to 0.20, slight agreement; 0.21 to 0.40, fair agreement; 0.41 to 0.60, moderate agreement; 0.61 to 0.80, good agreement; and 0.81 to 1.00, excellent agreement. A value of P < 0.05 indicated statistically significant difference.

The article "Clinical evaluation of new automatic coronary-specific best cardiac phase selection algorithm for single-beat coronary CT angiography" was published in 2017. Journal: PLoS One.

## Results

All scans were successfully completed in all of the 46 (22 male, 24 femal) enrolled patients. The average age was 58.4±11.3years; and age range was 31–78 years. The average heart rate was 91±18.5 bpm. The mean effective radiation dose was 1.34±0.52 mSv.

### Subjective evaluation of coronary arteries

A total of 204 vessels were evaluated. The overall inter-observer agreement for image quality scoring was moderate (κ = 0.68). The mean subjective image quality of the SP phase was comparable to that of the MS phase, 1.45±0.85 vs 1.43±0.81, respectively (p = 0.88). There were 9 (4.4%) non-diagnostic coronary vessels using the SP phase, vs 10 (4.9%) when using the MS phase with no significant difference between the two algorithms (p = 0.5). The subjective image quality scores are shown in Fig 1. There were also no difference of the individual coronary arteries between the two groups. The average image quality of RCA, LAD, LCX were shown in Table 1.

**Fig 1:** Comparison of subjective image quality of MS and SP phases. MS = Manual Selection, SP = Smart Phase. Image quality score: 1 = excellent, 2 = good, 3 = intermediate, 4 = poor.

**Table 1:** The average image quality of individual coronary arteries.

Vessel	Group	N	Average	SD	P
**RCA**	**SP**	**77**	**1.48**	**0.88**	**0.73**
	**MS**	**77**	**1.44**	**0.87**	
**LAD**	**SP**	**67**	**1.37**	**0.85**	**0.39**
	**MS**	**67**	**1.43**	**0.84**	
**LCX**	**SP**	**60**	**1.47**	**0.81**	**0.90**
	**MS**	**60**	**1.42**	**0.72**	

### Phase selection number and time

The mean numbers of reconstruction for SP were 13.55±5.03, while for the MS, these were 5.41±2.39 (p<0.01). However, the average reconstruction time of the SP was 97.81±26.71 s while the average reconstruction time of MS was 245.01±55.07 s, indicating that the SP used significantly less time (p<0.01) but reconstructed more phases. The average time savings were 148 seconds (60%). Fig 2 shows results of the number of reconstruction and time by these two groups. When the reconstruction increased, the reviewing time was significantly reduced with use of SP when compared to the MS.

**Fig 2:** Comparison of the numbers of reconstructions and time by MS and SP algorithms. MS = Manual Selection, SP = Smart Phase.

### The selected cardiac phase

The average best phase selected by SP was 48.26%±6.49%, while the average best phase determined by MS was 48.67%±7.16% with no significant difference between these two groups (p>0.05). Fig 3 shows the plots of selected cardiac phases using these two methods. For the heart rate between 80 bpm to 95 bpm, MS tends to select the phase from 42%-56%, however, the phases determined by SP were more scattered. Fig 4 shows the Box plot of phase reconstructions using different reconstruction strategies. No statistical difference was found between SP and MS methods (p>0.05). The center of the two methods were almost the same, while the range of SP group was larger. Fig 5 shows phase differences between the two groups. There was no statistic difference between the two groups. While the average absolute difference between SP and MS best phases was 2.29%±2.47%.

The article "Clinical evaluation of new automatic coronary-specific best cardiac phase selection algorithm for single-beat coronary CT angiography" was published in 2017. Journal: PLoS One.

**Fig 3:** Plots of selected cardiac phases. Distribution of selected cardiac phases with the use of MS and SP methods. MS-manual selection, SP-smart phase.

**Fig 4:** The box plot of phase reconstructions. The center phase of the two groups were almost overlap, but the SP group were more scatted than the MS group.

**Fig 5:** Differences in the selected phases. There was no statistic difference between the two groups.

## Discussion

Our results indicate that the phase selection algorithm that we evaluated can provide equivalent image quality to the MS but can also eliminate the reviewing time (despite having slightly longer reconstruction time). It may help the less experienced users to pick up the most suitable reconstruction phase when interpreting CCTA images. Even for the experienced users, it can save time and improve the workflow on the single beat CCTA examination with more efficiency.

The new generation of 256 MDCT is equipped with a 16cm wide-area gemstone detector enabling whole-heart imaging in a single-beat without moving the scanner table. It has been reported that image quality could be improved in patients with a high heart rate when diagnosing coronary artery disease [10]. Ultralow-Dose contrast agent volume as well as effective radiation dose yields diagnostic CCTA image quality [11, 12]. However, clinical experience shows that it is a time-consuming process for radiologists to pick up the best phase with the least motion for reconstruction from the cardiac cycle, and for less experienced radiologists this would be even more difficult to determine the best phase. This is especially a challenge when imaging under higher heart rate conditions.

The phase selection algorithm we evaluated is based on coronary specific, quantitative image quality metrics. Based on the data that is acquired in the cardiac cycle, it searches each phase and each image slice within each phase to find the phase that maximizes objective metrics such as circularity and edge strength. This is different from other best phase algorithm which is based on the 4D motion map on dual source CT scanners. The algorithm for dual source CT allows for depiction of the motion along the patient z-axis during the entire cardiac cycle [13]. Young et al [14]compared image quality of 64-slice multi-detector CCTA using automated and manual multiphase methods for the determination of optimal phases for image reconstruction in patients with various mean heart rates. Their results indicated that the reconstruction based on manual absolute timing provides better image quality than that with automated optimal-phase selection software (PhaseXact; Toshiba Medical Systems, Tokyo, Japan) reconstruction techniques. However, authors didn't record the time of these two methods. Further they did not assess the workflow efficiency of each method.

The article "Clinical evaluation of new automatic coronary-specific best cardiac phase selection algorithm for single-beat coronary CT angiography" was published in 2017. Journal: PLoS One.

Results of this study indicate that the automatic coronary-specific best cardiac phase selection can provide comparable image quality while taking less time. These are several reasons for such improved performance. First, SP was based on quantitative image quality metrics, so it can make sure the best phase is selected. Second, the SP evaluates all vessels according to the averaged image quality to get the best phase. For the same patient, it can make sure that the diagnostic coronary artery branches can be picked up as much as possible. Third, the reconstruction intervals were 2% for the SP to insure it can choose the best phase, corresponding to more phases than MS, with reconstruction intervals being 5%.

The reconstruction intervals of the MS was set as 5%, because we use 5% as clinical routine. It can provide good image quality while using relatively less time. While for the SP, its reconstruction time was shorter than MS, so we choose 2% as the interval to make sure it can get good image quality. That's why the SP technique can get more phases than the MS technique. The percentage of unassessable vessels was MS (4.9%) VS SP (4.4%) with no significant difference. This means adopting SP to determine the best phase for image reconstruction may lead to a high frequency of obtaining diagnostic CCTA images. The mean frequency of unassessable segments was 4% when using 64-sliceCT with a common approach to select phases for reconstruction of the CCTA images [15], indicating the consistency of our findings with the literature.

SP is more beneficial due to using less time while offering more efficient workflow. At lower heart rates, it is often the case that a single phase in diastole will be sufficient for diagnostic assessment. However, as heart rate increases, such as in our study cohort, the best phase may be either in systole or diastole and may require some searching to identify if done manually [16], which means more phases will be reconstructed as the heart rate increases. This is also confirmed by findings in this study.

The article "Clinical evaluation of new automatic coronary-specific best cardiac phase selection algorithm for single-beat coronary CT angiography" was published in 2017. Journal: PLoS One.

It has been reported that CCTA performed on the 256-slice CT scanner yielded significantly better image quality in patients with high HR [10, 17]. Long reconstruction time may be an obstacle of the single one-beat CCTA examination, especially in the heart center with large patient volume. Thus, SP fills in this gap. This study also reveals that phases determined by SP were more scattered, especially for the heart rate between 80 and 95 bpm, while the MS tends to select the phase from 42%-56%. On the one hand, the radiologists tend to pick up the phases of image sharpness in end-systole based on personal experiences in patients with high heart rate [18]. And for the MS, it would pick up the best phase from all reconstructed phases, which will insure the image quality, on the other hand, it may be attributable to the fact that MS in our practice the interval was 5% increments, while the SP interval was 2%, it will provide more optional phases. However, there was no statistic difference in the image quality between these two groups, possibly due to small number of patients included in this study.

## Limitations

First, we only include the high heart rate patients, so the efficiency of the SP in the low heart rate patients still needs to be verified. Second, we did not use this reconstruction method on the snapshot freeze technique, which will improve the image quality within the single-beat coronary angiography [19, 20], as this study mainly focused on the comparison of SP and MS. Third, diagnostic accuracy of CCTA with use of the SP approach were not evaluated, further studies will be needed to investigate it.

## Conclusions

The smart phase improves clinical workflow in high heart rate patients and provides similar image quality compared with manual cardiac best phase selection. Reconstruction of single-beat CCTA exams with SP can benefit the users with less experienced in CCTA image interpretation.
